# High CASC expression predicts poor prognosis of lung cancer: A systematic review with meta-analysis

**DOI:** 10.1371/journal.pone.0292726

**Published:** 2024-04-04

**Authors:** Hao Han, Huan Huang, An-ping Chen, Yang Tang, Xin Huang, Cheng Chen

**Affiliations:** 1 Department of Thoracic Surgery, The Affiliated Hospital of Zunyi Medical University, Zunyi, Guizhou, China; 2 Department of Thoracic Surgery, People’s Hospital of Dongxihu District, Wuhan, Hubei, China; Xiangya Hospital Central South University, CHINA

## Abstract

**Background:**

The long non-coding RNA cancer susceptibility candidate (CASC) has abnormal expression in lung cancer tissues and may correlate with lung cancer prognosis. This study aimed to comprehensively evaluate the association between CASC expression and the cancer prognosis.

**Methods:**

PubMed, Embase, Web of Science, Google Scholar, Cochrane Library, and China National Knowledge Infrastructure databases were searched until April 1, 2023, to obtain the relevant literature. Studies that met the predefined eligibility criteria were included, and their quality was independently assessed by 2 investigators according to the Newcastle-Ottawa Scale (NOS) score. Detailed information was obtained, such as first author, year of publication, and number of patients. Hazard ratio (HR) with a 95% confidence interval (CI) was extracted and grouped to assess the relationship between CASC expression and cancer prognosis. The dichotomous data was merged and shown as the odds ratio (OR) with a 95% CI was extracted to assess the relationship between CASC expression and clinicopathological parameters.

**Results:**

A total of 12 studies with 746 patients with lung cancer were included in the meta-analysis. The expression levels of lncRNA CASC2 and CASC7 were decreased, while those of CASC9, 11, 15, and 19 were induced in lung cancer tissues compared with paracancerous tissues. In the population with low CASC expression (CASC2 and CASC7), high CASC expression indicated a good lung cancer prognosis (HR = 0.469; 95% CI, 0.271–0.668). Conversely, in the population with high CASC expression (CASC9, 11, 15, and 19), high CASC expression predicted a poor lung cancer outcome (HR = 1.910; 95% CI, 1.628–2.192). High CASC expression also predicted worse disease-free survival (DFS) (HR = 2.803; 95% CI, 1.804–6.319). Combined OR with 95% CI revealed an insignificant positive association between high CASC expression and advanced TNM stage (OR = 1.061; 95% CI, 0.775–1.454), LNM (OR = 0.962; 95% CI, 0.724–1.277), tumor size (OR = 0.942; 95% CI, 0.667–1.330), and histological grade (OR = 1.022; 95% CI, 0.689–1.517).

**Conclusion:**

The CASC expression levels negatively correlate with lung cancer prognosis. Therefore, CASC expression may serve as a prognostic marker and a potential therapeutic target for lung cancer.

## 1 Introduction

Cancer is currently the top threat to global public health, imposing a heavy economic burden on the health system every year [1]. According to the 2021 World Cancer Statistics Report, approximately 19.8 million new cancer cases are expected worldwide in 2020, with cancer deaths approaching 10 million [2]. Compared with other cancers, lung cancer incidence and death toll rank first among men and third among women. The primary treatment for lung cancer is surgery combined with radiotherapy and chemotherapy [3, 4] and can be combined with targeted therapy or immunotherapy to boost efficacy. Although these therapies increase the 5-year survival rate of the disease, its prognosis remains poor [5, 6]. Moreover, since some treatment methods have entered the bottleneck period, cancer research has refocused on discovering novel approaches using molecular biology [7]. Many small molecules and compounds are involved in the occurrence and development of cancer and often investigated for finding new therapeutic targets and prognostic markers [8].

Long non-coding RNAs (lncRNAs) are associated with the occurrence and development of tumors [9]. These RNAs are more than 200 nucleotides long, have no protein-coding ability, and regulate gene expression by directly acting on downstream genes or signaling pathways [10]. They can also act as competitive endogenous RNAs that sponge and down-regulate microRNAs, indirectly regulating the expression of downstream targets [11] and affecting tumor cell proliferation, migration, invasion, and apoptosis [12, 13]. For example, Gu et al. reported that NNT antisense RNA 1 (NNT-AS1) may facilitate the proliferation, migration, and invasion of cholangiocarcinoma cells by enhancing epithelial-mesenchymal transition (EMT) via up-regulating E-cadherin and down-regulating N-cadherin [14]. Chen et al. revealed that small nucleolar RNA host gene 8 (SNHG8) promotes the proliferation of non-small-cell lung cancer (NSCLC) cells by increasing the expression of cyclin D1 (CCND1) and cyclin dependent kinase 6 (CDK6) via sponging and down-regulating miR-542-3p [15].

Among lncRNAs, those from the lncRNA cancer susceptibility (CASC) gene family are typically deregulated in lung cancer [16]. Abnormally expressed CASCs regulate the occurrence and development of the disease by affecting the proliferation, migration, invasion, and cisplatin resistance of lung cancer cells [17]. Thus, mounting studies attempt to explore the correlation between CASC expression and lung cancer prognosis [18]. However, because various CSACs have different expression levels in lung cancer, these studies are biased due to the small sample size, yielding contradictory results. Because of these shortcomings, a systematic review and meta-analysis were conducted in this study to determine whether a correlation exists between CASC expression and lung cancer prognosis.

## 2 Materials and methods

### 2.1 Search strategy

In line with the reporting guidelines of the Preferred Reporting Items for Systematic Reviews and Meta-Analyses (PRISMA) [19], 6 public electronic databases were browsed to obtain the suitable publications: PubMed, Embase, Web of Science, Google Scholar, Cochrane Library, and China National Knowledge Infrastructure. The related subject headings and search terms were as follows: “long non coding RNA cancer susceptibility,” “lnc RNA cancer susceptibility,” “cancer susceptibility,” “lncRNA CASC,” “lncCASC,” or “CASC,” and “Lung cancer,” “NSCLC,” “SCLC,” or “Lung adenocarcinoma.” The search also covered the references of the included articles. The search time was from the establishment of the database to April 1, 2023.

### 2.2 Inclusion and exclusion criteria

The included literature met the following criteria:

1. The research mainly explored the correlation between CASC expression and lung cancer prognosis.
2. Patients with lung cancer were divided into the CASC high expression group and low expression group based on RT-qPCR results.
3. A comprehensive detection method assessed the CASC expression levels in tumor tissue.
4. The study provided sufficient and usable data for evaluation.

The exclusion criteria were as follows:

1. The study data were insufficient or could not be evaluated.
2. The correlation between CASC expression and lung cancer prognosis was unevaluated.
3. The literature was a conference abstract, meta-analysis, or duplicate publication.
4. The study researched animals.

### 2.3 Quality assessment of included literature

Two researchers independently estimated the quality of included studies based on the Newcastle-Ottawa Scale (NOS) score. This scale evaluates primary studies through 3 modules and 8 items and involves the selection of the study population, comparability, and exposure/outcome evaluation [20]. It adopts the semi-quantitative principle of the star system to assess the literature quality; the higher the score, the higher the quality of the research. Comparability was rated up to 2 stars, while the other items were up to 1 star. The full score was 9 stars. Studies with a score of no less than 6 were thought suitable for inclusion in the meta-analysis.

### 2.4 Extraction of relevant data

Two researchers independently extracted the data of the included studies as follows: first author, publication year, number of patients, cut-off value, survival outcome, and hazard ratio (HR) value with 95% confidence interval (CI). If a survival curve was provided without HR and its 95% CI, the Engauge Digitizer software (v. 4.0) was employed to extract the HR value from the survival curve [21]. In addition, clinicopathological parameters were obtained: TNM stage, lymph node metastasis (LNM), distance metastasis (DM), tumor size, histological grade, depth of invasion, and patient age and gender. If the extracted data were inconsistent, they were judged through discussion or consulting a third researcher.

### 2.5 Ethics approval

This was a clinical retrospective analysis and requires no ethical statement.

### 2.6 Statistical analysis

The RevMan software version 5.4.0 (Cochrane Collaboration, London, UK) and STATA version 12.0 (StataCorp LLC, College Station, TX) were utilized for statistical analyses. Hazard ratio values with 95% CIs were pooled to assess the relationship between CASC expression and survival prognosis of NSCLC. The dichotomous data were merged and presented as odds ratio (OR) and 95% CI to explore the association between CASC expression and the clinicopathological parameters. For the heterogeneity, a random-effect model was applied, and subgroup analysis was conducted for high heterogeneity (*I*^*2*^ > 50, *P* < 0.05), while a fixed-effect model was adopted for low heterogeneity (*I*^*2*^ ≤ 50, *P* ≥ 0.05). Results with *P* ≤ 0.05 were considered statistically significant. The sensitivity analysis based on the STATA software was performed to explore the influence of data from individual studies on the overall results. The publication bias based on Begg’s test was conducted to reveal potential bias.

## 3 Results

### 3.1 The basic characteristics of the included literature

Based on the subject headings, 6 electronic databases were searched exhaustively, and 342 original studies were initially obtained. Among them, 68 were excluded because of duplication and 241 due to an unevaluated correlation between CASC expression and lung cancer prognosis. The other excluded studies were 5 meta-analyses, 8 reviews, and 8 articles with insufficient data. The 12 remaining available articles containing data from 746 patients were included in this study (Fig 1 and Table 1). All patients were Chinese and showed down-regulated CASC2 and CASC7 in lung cancer tissues [16, 17, 22, 23] but up-regulated CASC9, 11, 15 and 19 [18, 24–30]. Of the 12 included studies, all received an NOS scale score of no less than 6 points and were confirmed suitable for this study (Table 2).

**Fig 1:** The flow diagram of the eligible studies.

**Table 1:** Basic features of the publications included in this meta-analysis (n = 12).

author and year	sample size	lncRNA	expression level	cut-off value	survival outcome	HR with 95%CI	analysis method	source of HR value	follow-up month	NOS score
Xiao XH 2020	85	CASC2	downregulated	mean	OS	0.6 (0.36–1.01)	univariate analysis	survival curve	60	8
He XZ 2016	76	CASC2	downregulated	median	OS	0.276 (0.099–0.768)	multivariate analysis	paper	60	9
Tong LF 2019	86	CASC2c	downregulated	not reported	not reported	-	-	-	-	6
Chen L 2020	80	CASC7	downregulated	mean	OS	0.54 (0.28–1.04)	univariate analysis	survival curve	60	8
Zhao WG 2020	43	CASC9	upregulated	median	OS	1.78 (0.78–4.08)	univariate analysis	survival curve	60	8
Bing ZX 2021	40	CASC9	upregulated	median	OS	1.59 (0.59–4.28)	univariate analysis	survival curve	60	8
Zhang XD 2020	48	CASC9	upregulated	mean	OS	3.805 (1.4001–10.3407)	univariate analysis	survival curve	60	8
Fu Y 2019	71	CASC11	upregulated	mean	OS	2 (1.13–3.52)	univariate analysis	survival curve	60	8
Yan RC 2019	40	CASC11	upregulated	mean	OS	1.74 (0.76–3.99)	univariate analysis	survival curve	60	8
Li M 2019	95	CASC15	upregulated	mean	OS	1.901 (1.704–2.319)	multivariate analysis	paper	60	9
					DFS	2.803 (1.804–6.319)	multivariate analysis	paper	60	9
Bai Y 2019	52	CASC15	upregulated	mean	OS	3.34 (1.3–8.59)	univariate analysis	survival curve	60	6
Qu CX 2019	30	CASC19	upregulated	mean	OS	2.23 (0.72–6.88)	univariate analysis	survival curve	60	6

**Note:** CASC, cancer susceptibility candidate; OS, overall survival; HR, hazard ratio; CI, confidence interval; NOS, Newcastle-Ottawa Scale.

**Table 2:** Quality assessment of eligible studies Newcastle-Ottawa Scale (NOS) score.

Author	Country	Selection				Comparability	Outcome			Total
		Adequate of case definition	Representativeness of the cases	Selection of Controls	Definition of Controls	Comparability of cases and controls	Ascertainment of exposure	Same method of ascertainment	Non-Response rate	
Xiao XH 2020	China	*	*	*	*	*	*	*	*	8
He XZ 2016	China	*	*	*	*	**	*	*	*	9
Tong LF 2019	China	*	*	*	*	*	-	*	-	6
Chen L 2020	China	*	*	*	*	*	*	*	*	8
Zhao WG 2020	China	*	*	*	*	*	*	*	*	8
Bing ZX 2021	China	*	*	*	*	*	*	*	*	8
Zhang XD 2020	China	*	*	*	*	*	*	*	*	8
Fu Y 2019	China	*	*	*	*	*	*	*	*	8
Yan RC 2019	China	*	*	*	*	*	*	*	*	8
Li M 2019	China	*	*	*	*	**	*	*	*	9
Bai Y 2019	China	*	*	*	*	*	*	-	-	6
Qu CX 2019	China	*	*	*	*	*	*	-	-	6

### 3.2 The association between CASC expression and survival outcome

Among the 12 studies included in the meta-analysis, 11 with 660 patients assessed the relationship between CASC expression and overall survival (OS) of patients with lung cancer. The combined HR with 95% CI showed an insignificant positive relation between elevated CASC expression and poor OS of patients with lung cancer (HR = 1.272; 95% CI, 0.686–1.858) (Fig 2). High heterogeneity (*I*^*2*^ = 85.8; *P* < 0.0001) was also discovered; in lung cancer tissues with low CASC expression (CASC2 and CASC7), high expression of the transcript indicated a good prognosis of lung cancer. Conversely, in lung cancer tissues with high CASC expression (CASC9, 11, 15, and 19), high CASC expression predicted a poor prognosis. Based on the CASC expression levels in lung cancer tissues, a subgroup analysis was conducted, revealing that in the subgroup with high CASC expression, increasing transcript expression demonstrated poor prognosis (HR = 1.910; 95% CI, 1.628–2.192), while in the subgroup with low CASC expression, rising transcript expression predicted satisfactory prognosis (HR = 0.469; 95% CI, 0.271–0.668). A subgroup analysis was also performed based on analytical methods, HR extraction methods and cut-off value, showing that the CASC expression levels had no significant correlation with lung cancer prognosis. Finally, the last of the 12 studies evaluated the association between CASC expression and disease-free survival (DFS) in patients, uncovering that increasing CASC expression indicated poor DFS (HR = 2.803; 95% CI, 1.804–6.319) (Table 3).

**Fig 2:** Forest plot showing the relationship between CASC expression and overall survival (OS) of patients with lung cancer. **Note:** HR, hazard ratio; CI, confidence interval.

**Table 3:** Combined HRs of overall survival of patients with increased CASC expression.

Subgroup analysis	No. of studies	No. of patients	Pooled HR (95% CI)		*P*	Heterogeneity	
			Fixed	Random		*I* ^*2*^ *(%)*	*P-value*
**OS**	11	660	0.947 (0.784–1.109)	1.272 (0.686–1.858)	< 0.0001	85.8	< 0.0001
**CASC expression**							
High expression	8	419	1.910 (1.628–2.192)	1.910 (1.628–2.192)	< 0.0001	0	0.981
Low expression	3	241	0.469 (0.271–0.668)	0.469 (0.269–0.670)	< 0.0001	1.8	0.361
**Cut-off value**							
median	3	159	0.374 (0.051–0.697)	0.941 (-0.171–2.054)	0.097	58.2	0.091
mean	8	501	1.141 (0.953–1.329)	1.422 (0.712–2.132)	< 0.0001	85.9	< 0.0001
**HR statistics**							
Direction	2	171	1.157 (0.930–1.383)	1.090 (-0.503–2.682)	0.18	98	< 0.0001
Indirection	9	489	0.723 (0.490–0.957)	1.080 (0.600–1.561)	< 0.0001	44.8	0.070
**Analysis method**							
Multivariate analysis	2	171	1.157 (0.930–1.383)	1.090 (-0.503–2.682)	0.18	98	< 0.0001
Univariate analysis	9	489	0.723 (0.490–0.957)	1.080 (0.600–1.561)	< 0.0001	44.8	0.07
**NOS score**							
9	2	171	1.157 (0.930–1.383)	1.090 (-0.503–2.682)	0.18	98	< 0.0001
less than 9	9	489	0.723 (0.490–0.957)	1.080 (0.600–1.561)	< 0.0001	44.8	0.07
DFS	1	95	2.803 (1.804–6.319)	2.803 (1.804–6.319)	NA	NA	NA

**Note:** CASC: Cancer Susceptibility Candidate; OS: overall survival; HR: hazard ratio; CI: confidence interval; NOS, Newcastle-Ottawa Scale; *P*, statistical significance of the results; *P-value*, statistical significance of heterogeneity; *I*^*2*^, I-square.

### 3.3 The association between CASC expression and TNM stage

The meta-analysis investigated 8 studies with 507 patients to evaluate the association between CASC expression and the TNM stage. The combined OR with 95% CI predicted the insignificant positive relationship between high CASC expression and advanced TNM stage (OR = 1.061; 95% CI, 0.775–1.454) (Fig 3). Based on the CASC expression levels, the patients were assigned into a CASC low expression subgroup (CASC2 and CASC7) and a high expression subgroup (CASC9, 11, 15, and 19). In the high subgroup, increasing CASC expression indicated a poor lung cancer prognosis (OR = 1.745; 95% CI, 1.121–2.7189), whereas, in the low subgroup, rising CASC expression predicted a good prognosis (OR = 0.597; 95% CI, 0.371–0.960) (Table 4).

**Fig 3:** Forest plot depicting the relationship between CASC expression and lung cancer TNM stage. **Note:** OR, odds ratio; CI, confidence interval.

**Table 4:** Combined effects of clinicopathologic characteristics in patients with lung cancer exhibiting abnormal CASC expression.

Clinicopathologic characteristics	No. of studies	No. of patients	Odds ratio (95% CI)		*P*	Heterogeneity	
			Fixed	Random		*I*^*2*^(%)	*P*-value
**Age**	9	593	0.953 (0.721–1.258)	0.952 (0.720–1.258)	0.732	0	0.996
**gender**	9	593	0.954 (0.705–1.291)	0.953 (0.703–1.292)	0.761	0	0.967
**TNM** (**III**+**IV** vs. **I**+**II**)	8	507	1.061 (0.775–1.454)	1.095 (0.723–1.657)	0.711	37	0.134
CASC expression							
High CASC expression	5	266	1.745 (1.121–2.7189)	1.742 (1.117–2.715)	0.014	0	0.966
Low CASC expression	3	241	0.597 (0.371–0.960)	0.598 (0.371–0.962)	0.033	0	0.926
NOS score							
9	2	171	1.083 (0.590–1.987)	0.981 (0.282–3.407)	0.976	73	0.054
less than 9	6	336	1.054 (0.729–1.522)	1.111 (0.696–1.773)	0.658	32.4	0.193
**LNM (present vs. absent)**	8	550	0.962 (0.724–1.277)	0.961 (0.699–1.320)	0.787	16.1	0.304
CASC expression							
High CASC expression	4	223	1.439 (0.900–2.300)	1.420 (0.857–2.353)	0.128	9.7	0.345
Low CASC expression	4	327	0.753 (0.524–1.082)	0.753 (0.524–1.082)	0.125	0	0.897
NOS score							
9	2	171	1.348 (0.793–2.290)	1.335 (0.626–2.844)	0.269	49.4	0.16
less than 9	6	379	0.837 (0.597–1.173)	0.831 (0.590–1.170)	0.301	0	0.519
**Tumor size (big vs small)**	6	382	0.942 (0.667–1.330)	0.955 (0.602–1.513)	0.734	38.9	0.147
CASC expression							
High CASC expression	4	226	1.348 (0.847–2.145)	1.348 (0.843–2.158)	0.207	0	0.46
Low CASC expression	2	156	0.585 (0.342–1.002)	0.585 (0.342–1.002)	0.051	0	0.555
NOS score							
9	2	171	0.899 (0.538–1.503)	0.897 (0.285–2.823)	0.685	78.6	0.031
less than 9	4	211	0.979 (0.614–1.559)	0.984 (0.588–1.646)	0.927	13.2	0.326
**Histological grade**	5	284	1.022 (0.689–1.517)	1.020 (0.684–1.522)	0.913	0	0.524
CASC expression							
High CASC expression	3	128	1.525 (0.836–2.780)	1.523 (0.835–2.780)	0.169	0	0.932
Low CASC expression	2	156	0.742 (0.434–1.267)	0.742 (0.434–1.267)	0.274	0	0.991
NOS score							
9	1	76	0.739 (0.342–1.599)	0.739 (0.342–1.599)	0.443	NA	NA
less than 9	4	208	1.149 (0.724–1.822)	1.148 (0.719–1.833)	0.556	0	0.514
**DM (present vs. absent)**	1	80	0.406 (0.172–0.960)	0.406 (0.172–0.960)	0.04	-	-

**Note:** CASC, cancer susceptibility candidate; TNM stage, tumor, node, metastasis stage; LNM, lymph node metastasis; DM, distant metastasis; OR, odds ratio; CI, confidence interval; NOS, Newcastle-Ottawa Scale; *P*, statistical significance of the results; *P-value*, statistical significance of heterogeneity; *I*^*2*^, I-square.

### 3.4 The association between CASC expression and other clinicopathological parameters

The relationship between CASC expression and other clinicopathological parameters was also explored: LNM, DM, tumor size, histological grade, depth of invasion, age, and gender. An insignificant relation was revealed between high CASC expression and LNM (OR = 0.962; 95% CI, 0.724–1.277) (Fig 4), tumor size (OR = 0.942; 95% CI, 0.667–1.330) (Fig 5A), histological grade (OR = 1.022; 95% CI, 0.689–1.517) (Fig 5B), age (OR = 0.953; 95% CI, 0.721–1.258), and gender (OR = 0.954; 95% CI, 0.705–1.291) (Table 4).

**Fig 4:** Forest plot demonstrating the relationship between CASC expression and lung cancer LNM. **Note:** OR, odds ratio; CI, confidence interval.

**Fig 5:** Forest plot illustrating the relationship between CASC expression and lung cancer tumor size and histological grade. **Note:** OR, odds ratio; CI, confifence interval.

### 3.5 Sensitivity analysis and publication bias

Finally, Begg’s test was employed to conduct a sensitivity analysis and estimate publication bias. Removing the results of a single study would not significantly change the overall results, suggesting the data of this study have strong reliability and robustness (Fig 6). The test also showed that except for histological grade (Pr > |z| = 0.027), no significant publication bias among the various study outcomes was present, including OS (Pr > |z| = 0.938), the TNM stage (Pr > |z| = 0.174), LNM (Pr > |z| = 0.266), tumor size (Pr > |z| = 0.707), age (Pr > |z| = 1.000), and gender (Pr > |z| = 0.466) (Fig 7).

**Fig 6:** Sensitivity analysis for CASC expression with overall survival (OS) of patients with lung cancer. **Note:** HR, hazard ratio; CI, confifence interval.

**Fig 7:** Publication bias about the relationship between CASC expression and survival outcome in lung cancer. **Note:** (A) OS, overall survival; (B) TNM stage, tumor, node, metastasis stage; (C) LNM, lymph node metastasis; (D) Tumor size; (E) Histological grade; (F) Age; (G) Gender.

## 4 Discussion

Long non-coding RNAs are small molecules without protein-coding ability and were once considered uninvolved in the biological behavior of cells [31, 32]. As the research on diseases gradually moved focus from the individual to genes, many lncRNAs were discovered to participate in the progression of many diseases, such as cancer [33], cardiovascular [34], metabolic, and neurodegenerative diseases. Moreover, numerous ncRNAs have abnormal expression in cancer cells, affecting events detrimental to cancer prognosis, such as proliferation, migration, invasion, and apoptosis. For example, Chen et al. reported that long intergenic non-protein coding RNA 1234 (LINC01234) promotes the proliferation and migration and inhibits the apoptosis of gastric cancer cells by increasing core-binding factor subunit beta (CBFB) expression via sponging and down-regulating miR-204-5p [35]. Shi et al. demonstrated that long intergenic non-protein coding RNA 261 (LINC00261) hinders the proliferation, migration, and invasion of NSCLCs by suppressing the Wnt signaling pathway through sponging miR-522-3p [36].

The cancer susceptibility candidate family of lncRNAs contains dozens of cancer-related CASCs that promote or inhibit tumor progression by affecting cell proliferation, migration, invasion, and apoptosis [37]. Many researchers have tried to explore the correlation between CASC expression and cancer patients. However, due to the insufficient sample size of a single study and inconsistent conclusions among different studies, the reliability and robustness of the results are elusive. Therefore, this meta-analysis study was performed to determine the correlation between CASC expression and the prognosis of lung cancer.

Although combined HR value and 95% CI showed that high CASC expression predicted poor prognosis of lung cancer, this result was not statistically significant. Because of the inconsistent expression of different CASCs in lung cancer, we conducted a subgroup analysis and found that high CASC expression predicts poor prognosis of the disease. Furthermore, since the statistical methods differ among the included original articles (univariate analysis vs. multivariate analysis), follow-up time, source of HR value (paper vs. survival curve), and cut-off value, a certain degree of bias was present in the overall results. To reduce the bias, we conducted a subgroup analysis and showed that, in univariate or multivariate analysis subgroups, highly expressed CASC predicted poor prognosis of lung cancer. High CASC expression also predicted poor lung cancer prognosis in the mean and median subgroups. In addition, we evaluated the correlation of CASC expression levels with clinicopathological parameters of the patients. We demonstrated that high CASC expression correlated with the advanced TNM stage, low lymph node and distant metastases, large tumor diameter, and low pathological grade, conforming CASC expression is associated with the proliferation, migration, and invasion of tumor cells. Although our data show high CASC levels predict poor lung cancer prognosis, the underlying molecular mechanism remains unclear. Nonetheless, its missing steps are slowly uncovered by recent evidence (Fig 8). Xiao et al. revealed that CASC2 contributed to the proliferation, migration, and invasion of cisplatin-resistant NSCLCs cells (A549/DDP) by up-regulating interferon regulatory factor 2 (IRF 2) via sponging and suppressing miR-18a [16] (Table 5). Similarly, Tong et al. revealed that CASC2c facilitates the invasion, proliferation, and migration of colorectal cancer cells by activating the β-catenin signaling pathways [17]. He et al. demonstrated that CASC2 promotes the proliferation of NSCLCs but did not uncover the mechanism of this effect [22]. Other CASC members also affect different aspects of growth and metastasis of lung cancer cells. For instance, Chen et al. showed that CASC7 inhibits the proliferation and migration of NSCLCs by down-regulating N-cadherin and vimentin but up-regulating E-cadherin expression via sponging miR-92a [23]. Zhao et al. uncovered that CASC9 enhances the proliferation, migration, and invasion of NSCLCs by suppressing S100 calcium-binding protein A14 (S100A14) via sponging and down-regulating miR-335-3p [24]. Moreover, Bing et al. reported that CASC9 contributes to the proliferation and gefitinib resistance of NSCLCs by increasing forkhead box O3 (FOXO3) expression via interacting with miR-195-5p [25]. Yan et al. showed that CASC11 facilitates the proliferation, migration, and invasion of NSCLCs by regulating the expression of FOXO3 via sponging and suppressing miR-498 [18]. Furthermore, Li et al. demonstrated that CASC15 contributes to the migration, proliferation, and invasion of NSCLCs by activating epithelial-mesenchymal transition [28]. Bai et al. uncovered that CASC15 induces the invasion and proliferation of NSCLCs by up-regulating kallikrein related peptidase 12 (KLK12) expression through the down-regulation of miR-766-5p [29]. Qu et al. reported that CASC19 promotes the invasion, migration, and proliferation of NSCLCs by sponging and down-regulating miR-130b-3p [30]. Fu et al. uncovered that CASC11 may contribute to the stemness of small cell lung cancer cells by up-regulating TGF-β1 [27].

**Fig 8:** The lncRNA CASC has a critical biological role in lung cancer cells.

**Table 5:** The regulation mechanism of lncRNA CASC in lung cancer.

lncRNA	expression level	role	miR-RNA	gene or pathway	cell lines	function (high expression)	reference (PMID)
CASC2	downregulated	tumor suppressor gene	miR-18a	ELF1	H226, H520, SK-MES-1, A549, H1975, H1299, BEAS-2B	inhibits proliferation, migration, invasion and cisplatin resistance	32271431
CASC2	downregulated	tumor suppressor gene	-	-	A549, PC-9, and NCI-H1299	inhibited cell proliferation	26790438
CASC2c	downregulated	tumor suppressor gene	-	ERK1/2 and β-catenin signaling pathways	H292, H226, H1975 and H460	suppress proliferation and migration	31300295
CASC7	downregulated	tumor suppressor gene	miR-92a	E-cadherin, N-cadherin, Vimentin	A549, H358 and H2170	inhibits proliferation, migration and invasion	32626930
CASC9	upregulated	oncogene	miR-335-3p	S100A14	A549, H1299 and BEAS-2B	induce proliferation, migration, and invasion	32606808
CASC9	upregulated	oncogene	miR-195-5p	FOXO3	PC9/GR, H460, H1299, A549	enhances proliferation and gefitinib resistance	34619168
CASC9	upregulated	oncogene	-	CDC6	H1650, H460, SPC-A1 and A549	enhace proliferation, migration and cell cycle	33061598
CASC11	upregulated	oncogene	-	TGF-β1	SHP-77, H345 and H341	increased the stemness of SHP-77 and DMS 79 cells	30965130
CASC11	upregulated	oncogene	miR-498	FOXO3	A549, H460, H1299, H322	promote proliferation and cell cycle progression	31537383
CASC15	upregulated	oncogene	-	E-cadherin, N-cadherin, Vimentin	H1703, A549, SPC_x005f A1, NCI-H460 and NCI-1650	facilitate cell proliferation, migration and invasion	31396336
CASC15	upregulated	oncogene	miR-766-5p	KLK12	A549, H1299, H1975 and SPC-A-1	contributes to proliferation and invasion	31378128
CASC19	upregulated	oncogene	miR-130b-3p	ZEB2	A549, H322, PC9, and GLC-B2	promotes the proliferation, migration and invasion	31389608

**Note:** ELF1, E74-like factor 1; ERK, extracellular signal-regulated kinases; S100A14, S100 calcium binding protein A14; FOXO3, forkhead box O3; CDC6, cell division cycle 6; KLK12, kallikrein related peptidase 12; ZEB2, zinc finger E-box binding homeobox 2.

This study has several shortcomings. The patients included in this study were Chinese, making the conclusions applicable only to China or Asia. In addition, the sample size included in this study was not large, rendering the results and conclusions prone to selection bias. Another drawback is that although some included studies specified the HR value and 95% CI, others only provided the survival curve, necessitating indirect calculation of HR and resulting in the overall HR value being prone to statistical bias. Most CASCs were highly expressed in lung cancer tissues, and high CASC expression predicted poor survival outcomes in these subgroups. However, some CASCs were down-regulated in lung cancer tissues, and low expression of these transcripts predicted poor survival outcomes in these subgroups. Therefore, subgroup analysis was performed based on the expression level of CASC in this study. Despite the above limitations, this study has many advantages. It is the first meta-analysis to explore the correlation between the expression level of the CASC family and lung cancer prognosis. It showed by summarizing a large amount of data that high CASC expression predicts poor survival outcomes in lung cancer with high reliability and robustness. This study comprehensively summarized all the possible molecular mechanisms by which CASC affects lung cancer progression, providing a valuable reference for cancer treatment. It also provided a detailed subgroup analysis, comprehensively presenting the prognostic correlation between CASC expression and different subgroups and between CASC expression levels and various clinicopathological parameters.

## 5 Conclusion

Most CASCs are highly expressed in lung cancer and predict its poor prognosis. Thus, CASCs are potential therapeutic targets and promising prognostic markers in lung cancer.

## Supporting information

S1 Checklist PRISMA 2020 checklist. (DOCX)
